# Q-Switched Laser Combined with Intense Pulsed Laser in the Treatment of Melasma Based on Reflection Confocal Microscope

**DOI:** 10.1155/2022/4413130

**Published:** 2022-07-01

**Authors:** Jiali Xu, Yijing Pu

**Affiliations:** Tonglu County First People's Hospital, Zhejiang Hangzhou, Tonglu 311500, China

## Abstract

Chloasma is a prevalent clinical hyperpigmentation skin disorder that causes symmetrical brown to tan patches on the cheeks, as well as the neck and forearms on rare occasions. The pathophysiology of this condition is complicated, and there is now no cure. Under the light microscope, the full-thickness melanin of the epidermis in the skin lesions was increased, and the dermal chromophages increased. At present, the treatment of melasma mainly includes topical drugs, chemical peels, systemic drugs, laser therapy, and traditional Chinese medicine. With the development of medical technology, intense pulsed light and Q-switched laser have been widely used in the treatment of melasma, which can emit laser beams to penetrate the dermis uniformly to treat deep pigmented lesions in the dermis. After a stable treatment outcome for melasma is achieved, it is important to minimize side effects such as postinflammatory hyperpigmentation and skin irritation. Therefore, this paper uses a reflection confocal microscope to establish an evaluation index system and then uses a neural network to evaluate the treatment effect. The work of this paper is as follows: (1) this paper introduces various methods of treating melasma at home and abroad and focuses on the application of intense pulsed light therapy and low-energy Q-switched Nd: YAG laser in the treatment of melasma. (2) In this paper, the case data samples are trained with the designed BP network to obtain a reliable evaluation network model. (3) The results and mistakes of the evaluation are produced by training the genetic algorithm optimized backpropagation (GA-BP) network structure model to evaluate the treatment effect of chloasma. Finally, it has been demonstrated that the GA-BP network has great accuracy and stability.

## 1. Introduction

Chloasma is a pigmented skin disease. The pigmented spots are usually light brown or dark brown and distributed symmetrically on the cheekbones, forehead, and eyebrows and around the eyes and can also involve the dorsum of the nose, the alars of the nose, and the upper lip and lower whiskers. The border of the stain is clear or diffuse, the surface is free of inflammatory dandruff and flat to the skin surface, and most patients do not have any symptoms. Chloasma is more common in young and middle-aged women with darker skin and less common in men. Modern medicine believes that the pathogenesis of chloasma is extremely complex, and the latest research shows that the formation of chloasma may be related to local inflammation. Chloasma is characterized by an increase in melanin in the basal layer and acanthus layer of the epidermis, the number of melanocytes is normal or increased, the cell body is enlarged, the dendrites are obvious, and pigmented disease is characterized by histological features of free melanin granules in the upper dermis or phagocytosis by melanophagocytes. UV rays, hereditary factors, endocrine factors, cosmetics, uterine and ovarian illnesses, hepatitis A and B, oral contraceptives, and phototoxic medicines are the most common causes of chloasma. UV radiation, hereditary factors, endocrine factors, and cosmetics are the most important among these factors [1]. At present, the methods of treating melasma mainly include topical depigmentation agents, oral drugs, chemical peeling, and traditional Chinese medicine treatment. In recent years, technologies such as laser, intense pulsed light, microneedle introduction, and radio frequency technology have been increasingly applied to the treatment of melasma, and good results have been achieved [2]. Intense pulsed light is a broad-spectrum light in the 500-1200 nm band. According to selective photothermolysis theory, the pigment agglomeration preferentially absorbs laser energy after being irradiated with a specific wavelength of laser light, which can cause a blasting effect quickly, and then changes. The superficial ones are excreted with the skin flakes, and the deep ones are transported away with the lymphatic/blood circulation, so that they can be used to treat pigmented diseases [3]. However, the absorption of light by melanin is not limited to a single wavelength: in the wavelength range of 500-1200 nm, structures containing melanin can absorb the energy of light and cause photothermal decomposition [4]. However, since melasma melanocytes are unstable, it is an unstable disease, and any stimulation may aggravate the melasma, so the treatment of melasma needs to be gentle. The pulse width of the Q-switched laser is as short as nanoseconds, which is smaller than the thermal relaxation time of the melanin particles. The extremely high peak power can cause the melanin particles to be heated and exploded instantaneously. The treatment of sexually enhanced skin disease provides a new idea [5]. It avoids uneven distribution of energy, the treatment is relatively gentle, and the postoperative inflammatory response is mild. Therefore, the Q-switched ruby laser in the fractional mode is relatively safe for the treatment of melasma, and the incidence of side effects such as erythema, hyperpigmentation, and hypopigmentation is low [6]. In order to confirm the efficacy and safety of intense pulsed light and Q-switched laser in the treatment of melasma and to further explore its effects on melanocytes and melanin granules. In this paper, the RCM is used for postoperative observation. It has the characteristics of instant, noninvasive, and dynamic, and the detection depth can reach 300-500 *μ*m. The imaging resolution is high, and the epidermis and superficial dermis can be clearly observed. Then, use the neural network to analyze the obtained data, and finally, output the predicted value of the treatment effect of the Q-switched laser combined with the intense pulsed laser on melasma.

The application of intense pulsed light therapy and low-energy Q-switched Nd: YAG laser in the treatment of melasma is the emphasis of this paper, which introduces several methods of treating melasma at home and abroad. To obtain a reliable diagnosis and evaluation network model, the reliable diagnostic and evaluation case data samples are trained with the designed backpropagation neural network (BPNN) in this paper.

The paper arrangements are as follows: Section 2 describes the related work.  Section 3 defines the various methods.  Section 4 analyzes the experimental analysis.  Section 5 concludes the article.

## 2. Related Work

The pulse width of the Q-switched laser is nanoseconds. Since its wavelength is within the wavelength range absorbed by melanosomes and the pulse width is smaller than the thermal relaxation time of melanosomes, melanosomes selectively absorb light instantaneously. It can be raised to a very high temperature, and then, the melanin particles are smashed and disintegrated under the action of strong mechanical waves and are swallowed by macrophages, and the surrounding healthy tissues are not damaged. Q-switched laser is a classic laser for the treatment of pigmented diseases. There are many studies at home and abroad, but it also has a series of shortcomings, such as easy to cause pigmentation and hypopigmentation. Large-spot, low-energy, long-wavelength O-switched lasers have been utilized to treat pigmented illnesses in recent years to avoid the emergence of negative effects. The researchers applied a Q-switched fractional ruby laser with an energy of 2-3 J/cm^2^ to Asian female patients for 6 treatments at two-week intervals and concluded that a large-spot, low-energy Q-switched fractional ruby laser can effectively treat yellow for chloasma; from the histopathological point of view, the epidermal pigmentation was reduced after treatment, and the pigment content in the basal layer of the epidermis was reduced [7].

Reference [8] used the same kind of laser treatment, the energy was 4-8 J/cm^2^, and the subjects were all Caucasians, and the study showed that the treatment consequence was remarkable. However, its exact mechanism of action remains to be further explored. In addition, the high recurrence rate after laser treatment is an urgent problem to be solved. The curative effect of Q-switched 1064 nm laser and fractional 1064 nm laser was compared and it was concluded that there was no significant difference in the total effective rate of the two groups in the treatment of melasma, and the recurrence rate was low during the 1-year follow-up. Among them, the skin reaction after fractional 1064 nm laser treatment is mild, has less complication, has high comfort, and has a good application prospect. Reference [9] divided the subjects into 3 groups. The first group applied low-energy Nd: YAG laser once a week. The second group was treated with fruit acid once every 2 weeks, and the third group was treated with high-energy Nd: YAG laser once every 2 weeks. The results showed that the treatment effect of the first group was the best, followed by the second group, and finally the third group. Low-energy Nd: YAG laser is safe and effective in the treatment of melasma. Reference [10] treated melasma with a high-energy Nd: YAG laser, which resulted in increased pigmentation and new pigmentation. In reference [11], in order to explore the freckle removal mechanism of Nd: YAG laser, before treatment, after 5 times of treatment, and after 9 times of treatment, the pigmented skin was observed by an in vivo confocal microscope, which clearly and intuitively showed the mechanism of action. Strong light therapy for chloasma has been widely used in clinical practice. It is a broad-spectrum visible light with relatively concentrated wavelength and adjustable pulse width. The continuous wavelength is 500-1200 nm. Melanocytes in skin lesions selectively absorb some wavelengths of strong light. The photothermal effect is generated after the light is exposed, and it is broken and necrotic. The superficial pigment tissue is damaged and necrotic, and phagocytes phagocytose and expel the deep pigment. After severe light exposure to pigmentation, immediate deepening of the pigmentation and localized skin erythema appear. Strong light and Q-switched lasers were examined for their effectiveness in the treatment of melasma. Patients with melasma were treated using a combination of a bright light and a Q-switched laser. There was a statistically significant difference in the overall effectiveness of therapy between the bright light and Q-switch groups, but there was no significant difference in postoperative recurrence rates between the two groups, according to the data. Epidermal pigmentation and vascular disease can be effectively treated with bright light, although the impact on dermal pigmentation is minimal [12]

Treatment with the Q-switched Nd: YAG laser is the gold standard for chloasma; however, it is time unbearable and taxing on patients. Combining these two lasers to remove melasma can enhance the consequence. The experiment of reference [13] confirmed this point. The researchers first performed a bright light treatment on the subjects and then started the Q-switched Nd: YAG laser treatment two weeks later, a total of 4 times, with an interval of one week. The results showed that the curative effect was significant and the recurrence was effectively suppressed. It was concluded that the combination of the two and a single treatment was safe and effective with minimal adverse effects and that the Q-switched Nd: YAG laser paired with powerful pulsed light is worthy of promotion. Q-switched Nd: YAG laser and nonablative fractional 1550 nm laser were used for the treatment of freckles. Nonablative fractional laser was not found to have an auxiliary effect when Nd: YAG laser was used to treat melasma, and the effect of combined treatment was not significantly different from that of Nd: YAG laser treatment alone, according to the subjects [14]. Although laser treatment of melasma is effective, it also has different degrees of side effects. The recurrence rate of strong light therapy is relatively low, the recurrence rate of Q-switched laser is high, and it is easy to produce pigmentation. Fractional laser therapy has a high probability of postinflammatory pigmentation, and the pain is severe during treatment. In general, laser therapy is safer and more effective for light-skinned patients, but it should be used with caution in dark-skinned patients. With the introduction of new treatment theories and the emergence of new treatment instruments, laser treatment of melasma will become more and more important [15–18]. The organic and reasonable combination of various instruments will further improve the efficacy of the laser and reduce the side effects of laser treatment. Different pathological types and different skin types have different optimal responses to the instrument, and the optimal therapeutic parameters of various instruments for treating melasma in different periods are also different.

## 3. Method

This section discusses the BP neural network and defines the improvement of BP algorithm. They examine the treatment effect evaluation index system.

### 3.1. BP Neural Network

They discuss the establishment of the BP network model.

#### 3.1.1. BP Neural Network Model

The learning of the BP network in the ANN uses the error backpropagation algorithm, which is one of the most mature and perfect artificial neural networks at present. It is categorized by a simple structure and self-learning and parallel processing abilities; because it belongs to the classifier, it can form any decision-making area. The commonly used BP network is a three-layer structure. Forward propagation and backpropagation constitute the learning process of the BP network, each layer of the network has one or more neuron nodes, and the information is composed of the input layer which is passed to the output layer through each hidden layer, and the connection weight is used to represent the strength of the connection between the layers. The backpropagation learning method, or BP algorithm, may be used to alter the network's link weight such that the mapping relationship between the provided input and output of the network can be determined. There is no longer any room for mistake. The following relationship applies to the output layer:

(1) $$\begin{array}{c} O_{k}=f\left(neL_{k}\right),\;k=1,2,\cdots ,l, \end{array}$$

(2) $$\begin{array}{c} neL_{k}=\overset{m}{\underset{j=1}{\sum }}w_{jk}y_{j},\;k=1,2,\cdots ,l. \end{array}$$

For the hidden layer, there are the following relationships:

(3) $$\begin{array}{c} y_{j}=f\left(neL_{j}\right),\;j=1,2,\cdots ,m,\\ neL_{j}=\overset{n}{\underset{i=1}{\sum }}v_{ij}x_{j},\;j=1,2,\cdots ,m. \end{array}$$

In the above two formulas, let the transition number *f*(*x*) be a unipolar sigmoid function:

(4) $$\begin{array}{c} f\left(x\right)=\frac{1}{1+e^{-x}.} \end{array}$$

Formulas (1)–(4) together constitute the mathematical model of the three-layer perceptron.

#### 3.1.2. The Learning Process of the BP Network

The primary goal of the BP training procedure is to provide a certain input sample and get a specific output. Until a predefined error value is reached, the weights are modified based on the difference between the actual and predicted output values. The method is based on continuously modifying the threshold's weights and network parameters by propagating the error on one side and correcting the error on the other. For each training, it executes two propagation computations. The specific process is shown in Figure 1.

If the network output is not equal to the expected output, there will be an output error *E*, which is defined as follows:

(5) $$\begin{array}{c} E=\frac{1}{2}{\left(b-O\right)}^{2}=\frac{1}{2}\overset{l}{\underset{k=1}{\sum }}{\left(b_{k}-O_{k}\right)}^{2}. \end{array}$$

Expand the above error definition to the hidden layer; then,

(6) $$\begin{array}{c} E=\frac{1}{2}\overset{l}{\underset{k=1}{\sum }}{\left[b_{k}-f\left(\overset{m}{\underset{j=0}{\sum }}w_{jk}y_{j}\right)\right]}^{2}. \end{array}$$

Expanding further to the input layer, then

(7) $$\begin{array}{c} E=\frac{1}{2}\overset{l}{\underset{k=1}{\sum }}{\left\{b_{k}-f\left[\left(\overset{m}{\underset{j=0}{\sum }}w_{jk}f\left(\overset{m}{\underset{j=0}{\sum }}v_{ij}x_{i}\right)\right.\right]\right\}}^{2}. \end{array}$$

This shows that the network error depends on the weights of each layer; hence, modifying the weights may affect error. Adjusting the weights is a continuous process of reducing the error; hence, the weight adjustment should be proportionate to the error gradient:

(8) $$\begin{array}{c} ∆w_{jk}=\frac{-\mu^{\partial E}}{\partial w_{jk}},\;j=0,1,2,\cdots ,m,k=1,2,\cdots ,l,\\ ∆v_{ij}=\frac{-\mu^{\partial E}}{\partial v_{ij}},\;i=0,1,2,\cdots ,n,j=1,2,\cdots ,m, \end{array}$$

where − represents the gradient descent and the constant *n* belongs to the number between (0, 1).

#### 3.1.3. The Establishment of the BP Network Model

It is possible to choose the number of hidden layers and neurons at random in principle, but in practice, it is best to base this decision on the specifics of the problem at hand. For networks with a large number of hidden layers, training time is required since they are more likely to fall into a local minimum during training. After multiple testing, however, it was discovered that using a three-layer neural network was more accurate. Second, estimate the number of neurons in the output layer and input layer based on the data to be collected and the important elements influencing this layer as well as the feasibility of acquiring these influencing factor data. The hidden layer nodes may be identified without rules by counting the input and output nodes. Input nodes are the patient's important data, output nodes are the evaluation result, and hidden layer nodes can be identified without rules by counting the input and output nodes. The following formula may be used to determine the implicitly three-layer network according to the Kolmogorov theorem:

(9) $$\begin{array}{c} H=\sqrt{m+n}+a, \end{array}$$

where *H* represents the number of neurons in the hidden layer, *m* represents the number of neurons in the input layer, *n* is the number of neurons in the output layer, and *a* is a constant ranging from 1 to 10.

#### 3.1.4. Processing the Input Data of the BP Network

Due to the characteristics of the BP network itself, the selection of sample data has a great influence on the convergence speed and prediction accuracy. The saturation of the output function curve is caused by too large or too small input, so, in order to avoid the saturation area at both ends of the function and make the input play a strong role, it is necessary to normalize the input of the network. The formula for processing is as follows:

(10) $$\begin{array}{c} X=\frac{I-I_{\min}\;}{I_{\max}-I_{\min}}, \end{array}$$

where *I* represents the unprocessed neural network input value; *X* represents the smoothed neural network input value; and *I*_max_ and *I*_min_ are the maximum and minimum input values of the network input, respectively.

#### 3.1.5. Select the Learning Rate

Training weight changes are dictated by the learning rate: a low learning rate may lead to a lengthy training period and an inefficient convergence rate, while a high learning rate may cause the system to malfunction. As a result, a low learning rate is often used in order to maintain system stability. There is a choice of a learning rate ranging from 0.01 to 0.7. The learning rate of 0.2 is chosen in this study based on the actual training circumstances

### 3.2. Improvement of the BP Algorithm

Although the BP neural network has many remarkable features, it also has certain limitations: the hypersurface of multiple local minimum points constitutes the connection weight space formed by the global error *E* of the BP network, but the essence of the training method currently used by the BPNN is as follows: the method to search for the optimal connection weight in the connection weight space formed by the global error *E* is a point-to-point search. Because the network structure parameters at the start of the BPNN training are randomly assigned values, the BPNN cannot avoid slipping into a local minimum. Therefore, in the search process, it is very important to determine the position of the starting point. To eliminate the shortcoming that BPNN is easy to fall into local minima, it is necessary to improve the training method of BPNN, overcome the blindness and randomness of network structure parameters given at the beginning of network training, and let BPNN training start at the beginning. The weight falls on the global optimal peak area in the connection weight space formed by the global error *E*. When the BPNN is used for diagnosis and evaluation, the parameters of the obtained problem network model are easy to fall into local minima, and the network diagnosis and evaluation model cannot achieve satisfactory diagnosis and evaluation results every time, so it is necessary to improve the shortcomings of the BPNN that is easy to fall into local minima.

#### 3.2.1. Genetic Algorithms

Genetic algorithm (GA) is a global optimization algorithm. Its objective function does not need to be continuous or differentiable. It is different from the single-point search method in that it uses a method of parallel processing of multiple individuals in the search space. It has good global search performance and can effectively reduce the possibility of falling into local minima. It is mainly used in three aspects of neural network: optimization of connection weights, optimization of learning rules, and optimization of network structure, and the most important one is the weight of training neural network. In essence, genetic algorithms are used to replace some classic learning algorithms. The neural network's connection weights are where all of the system's knowledge is spread. Using a certain weight change rule is the traditional method to obtain the weights. The training process of the BPNN is as follows: continuously adjust the weights during training, and finally, get a good weight distribution, but if the training time is too long, it may fall into a local minimum value, so that a suitable weight distribution cannot be obtained. To solve this problem, GA can be used to optimize the connection weight. The process of combining GA and BP algorithm for neural network training is as follows: the algorithm parameters used in the training process are very sensitive to the results of BP algorithm and GA, and the result of BP algorithm is the same as the initial state of the network. At the beginning of the genetic algorithm, the optimal weight distribution range of the network is obtained by searching the weight space formed by the global error *E* of the BPNN, and then, the BP algorithm is used to find the optimal solution in the optimal weight distribution range. Finally, it is concluded that the combination of BP algorithm and GA is a feasible way for the hybrid training of neural network, and the combined algorithm is called GA-BP algorithm.

#### 3.2.2. Design of the GA-BP Algorithm

The main idea of using genetic algorithm to optimize the diagnosis and evaluation model of BPNN is as follows; based on BNN, the input and expected output of BPNN are normalized data. In this process, the BP algorithm is combined with the GA, and the gradient information of the BP algorithm, the advantages of strong local search ability, and the characteristics of the GA with high search efficiency and global search ability are used to train the neural network, so as to eliminate the BNN. In lattice training, the drawback is that it is simple to slip into the minimal value.  Figure 2 depicts the GA-functional BP's modules. It is made up of four essential components: input parameter preprocessing, output data restoration, neural network subfunction module, and GA-BPNN learning algorithm. The parameters of the grid model are continuously changed by training with known samples, and the model can be used to diagnose and evaluate the therapy effect of unknown disorders.

The stages of genetic algorithm optimization of neural network connection weight are as follows: (1) for a set of randomly generated distribution weights, for each weight (or threshold) in this group, use the coding scheme to encode, so as to build each code chain; for the case where the training rules and network structure have been determined, this code chain corresponds to a neural network whose weights and thresholds take specific values. (2) Calculate the neural network's error function and its fitness function value. The less fit you are, the greater the mistake you make. (3) Next generation inherits a fitness function value from the greatest person. (4) In order to create the next generation of organisms, genetic operators such as crossover and mutation are utilized. (5) Repeat the above process to continuously evolve the initially determined set of weight distributions until the training target meets the requirements.

#### 3.2.3. Implementation of GA-BP Algorithm Neural Network

(1) Coding of network structure parameters: the GA is used to improve the BP algorithm, but the network structure parameters are dry. Genetic operations cannot directly deal with it, so it is necessary to encode the network structure parameters before training to convert it into the genes of chromosomes composed of a certain structure. The real number encoding scheme and the binary encoding scheme are mostly these two procedures to encode the weights and thresholds in the network. Although the binary encoding is simple and common, its disadvantages are as follows: low precision, encoding strings is very long, and the real encoding scheme does not have this disadvantage; it is intuitive. There will be no situation of insufficient precision, and it needs a special genetic operation design for one-dimensional real numbers. This design chooses the real number coding scheme, which can speed up the evolution
(2) Select the fitness function: most of the genetic algorithm searches do not need external information, as long as the fitness function is used as the basis; the fitness value of each individual in the population is used to search. The fitness function used in this study is
  (11) $$\begin{array}{c} f=\frac{1}{E}, \end{array}$$
  where *E* is the global error. From formula (11), it can be known that the smaller the global error *E* is, the stronger the adaptability is
(3) Selection operator: evaluate each weight and threshold, and select the probability *P*_*i*_ as follows:
  (12) $$\begin{array}{c} P_{i}=\frac{f_{i}}{\sum_{i=1}^{m}f_{i}}, \end{array}$$
  where *f*_*i*_ represents the fitness value of the individual
(4) Crossover and mutation operation: these two factors have a great influence on the running performance of heredity, and a relatively small crossover rate is selected. And the mutation rate can increase the chance of individuals to transfer to the next generation. This choice is used for solutions with high ability, conversely, to eliminate solutions of individuals with low fitness ability. It is necessary to choose a relatively high crossover rate and mutation rate. The operation methods of the adaptive crossover rate *P*_c_ and mutation rate *P*_m_ used in this design are as follows:
  (13) $$\begin{array}{c} P_{\text{c}}=\frac{C}{f_{\max}-f_{a}},\\ P_{\text{m}}=\frac{d}{f_{\max}-f_{a}}, \end{array}$$
  where *c* and *d*  are constants less than 1, *f*_max_ is the maximum fitness value, and *f*_*a*_ is the average fitness value
(5) Determine genetic manipulation control parameters: mutation probability, crossover probability, and population size are three parameters to be controlled by the genetic algorithm. The setting of the values of these three parameters has a direct effect on the execution result of the genetic algorithm. For the size of the group; if the size is larger, the diversity of individuals in the group will be more, so although it is easy to find the global optimum, if it is too large, it will increase the calculation and cause the speed of finding the global optimum to be very slow. If the population size is too small, the search space range of the GA will be limited, which will lead to premature convergence. The population is estimated to be in the range of 20 to 100 people. The chosen group size is 20 since it meets the requirements of this design. If the crossover probability is very high, the individual structure of high fitness will be destroyed; if the crossover probability is too low, global search will be difficult. The crossover probability should, in general, be between 0.4 and 0.99; in this example, it is set to 0.5. For mutation operators, if the mutation probability is too high, the grid's evolutionary algorithm will fail, and the network will devolve into a pure random search; if the mutation probability is too low, new mutations will be difficult to generate

### 3.3. Treatment Effect Evaluation Index System

(1) MASI scoring method. According to the MASI international evaluation standard, the facial skin is divided into four areas, namely, the forehead, right cheek, left cheek, and mandible; the three indicators for evaluating the severity of skin lesions are skin lesion area percentage, color, and consistency of color distribution
  (14) $$\begin{array}{c} M=0.3\left[\left(DF+HF\right)AF+\left(D\text{MR}+\text{MR}\right)A\text{MR}+\left(D\text{ML}+H\text{ML}\right)A\text{ML}\right]+0.1\left(DC+HC\right)AC, \end{array}$$
  where *M* is MASI, *D* is color, *H* is consistency, *A* is area, *F* is forehead, MR is right cheek, ML is left cheek, and *C* is jaw.
  (15) $$\begin{array}{c} \text{MASI reduction rate}=\frac{V_{\text{b}}-V_{\text{a}}}{V_{\text{a}}}, \end{array}$$
  where *V*_b_ is value before treatment and *V*_a_ is value after treatment. See Table 1 for details.
(2) RCM scoring method. The laser beam scans from the spinous layer to the basal layer, mainly to observe the pigment density, cell brightness, and cell morphology; scans to the epidermis junction to observe the brightness of the pigment ring; and scans to the superficial dermis to observe inflammatory cells and melanocytes, elastic fibers, and blood vessels. Before treatment, the values were calculated after 2, 5, and 10 treatments. This experiment mainly observed 5 items of epidermal pigmentation density, number of dendritic cells and melanophages, elastic fibrosis, and vascular proliferation. The specific scoring standards are shown in Table 2

In this paper, the five indicators of RCM score are selected as input, and the treatment effect of four grades is used as output.

## 4. Experiment and Analysis

Here, the experimental results of BP algorithm are discussed, and the GA-BP algorithm experimental results are defined.

### 4.1. Experimental Results of the BP Algorithm

Valuable samples were formed through case records of dermatological patients in a tertiary hospital. From the 240 samples of reliably diagnosed cases, 200 were randomly selected as training samples and the remaining 40 as test samples. After 1000 iterations of BP neural network learning, the network performance target is set to 0.001, and the learning rate is set to 0.2. After training the BP network with the training samples, the test sample results are shown in Figure 3.

From the comparison error output in Table 3, it can be seen that most of the errors between the actual value of the patient's condition and the diagnostic value are not large, and one of the errors is large because a minimum value appears during network training. A small amount of error may be largely affected by the number of selected learning samples. In general, the construction and training of this BP network are feasible.

### 4.2. GA-BP Algorithm Experimental Results

The parameters of the genetic algorithm are selected as follows: the number of iterations is 40, the population size is 20, the crossover probability is 0.3, and the mutation probability is 0.01. First, randomly produce an initial population with an individual code length of 100; then, use the genetic algorithm to iterate 40 times to attain excellent individuals according to the modifications in the fitness function; decode the best individual found and assign it to the BP network; use the train function to train the network; and then, input the normalized test data into the trained network. Using the sim function for prediction, the normalized diagnostic values of 10 test samples will be obtained, which can be denormalized by mapminmax.  Figure 4 shows the fitness change curve when the genetic algorithm optimizes the neural network. It can be found from the figure that the 6th generation is a turning point of the fitness curve, from the initial fitness value of 55 to 30, indicating that after 6 generations of evolution, the GA-BP network has acquired better individuals.

It can be seen from Figure 5 that the optimized GA-BP network is superior to the traditional BPNN under the same training conditions. The output of the BPNN is always changing, and the output of the GA-BP network, on the other hand, is rather steady despite the outcomes of repeated tests. GA-BP network output is less volatile and stable compared to the classic BP. The BP network has an average error of 0.325, whereas the GA-BP network has an average error of 0.156. The GA-BP network is shown to be more accurate than the BP network. It can be seen from the above analysis that compared with the traditional BPNN, the use of the GA-BP network to establish a diagnostic model overcomes the inherent defects of the traditional BPNN and has the advantages of higher accuracy and better stability. Therefore, the GA-BP network can be used to evaluate the effect of laser treatment of melasma.

## 5. Conclusion

There are different forms of face pigment spots induced by various lasers, including chloasma, freckles, black spots, and sequelae, with chloasma being the most prevalent. Chloasma is a light brown to dark brown hyperpigmented skin illness with well-defined patches that are symmetrically distributed over the forehead, neck, around the eyes, around the lips, and other areas and vary in size and shape. It has no inflammatory manifestations, no dandruff, and no symptoms. Chloasma is more common in middle-aged persons, particularly women, and it lasts an average of 96.3 months. There are many ways to treat melasma: such as drug treatment, laser treatment, and Chinese medicine treatment. Among them, intense pulsed light therapy and low-energy Q-switched Nd: YAG laser have been widely used in the treatment of melasma, which can emit laser beams to penetrate the dermis uniformly to treat deep pigmented lesions in the dermis. After a stable treatment outcome for melasma is achieved, it is important to minimize side effects such as postinflammatory hyperpigmentation and skin irritation. Therefore, this paper uses RCM to establish an evaluation index system and then uses a neural network to evaluate the treatment effect. The work of this paper is as follows: (1) this paper introduces various methods of treating melasma at home and abroad and focuses on the application of intense pulsed light therapy and low-energy Q-switched Nd: YAG laser in the treatment of melasma. (2) In this paper, the reliable diagnosis and evaluation case data samples are trained with the designed BPNN to obtain a reliable diagnosis and evaluation network model. (3) By training the GA-BP network structure model to evaluate the treatment effect of chloasma, the results and errors of the evaluation are obtained. Finally, it is proved that the GA-BP network has the advantages of high precision and good stability, so it can be used to evaluate the effect of laser treatment of melasma.

## Figures and Tables

**Figure 1:** Network error definition and weight adjustment ideas.

**Figure 2:** GA-BP neural network model structure diagram.

**Figure 3:** When the training curve is 138 steps, the convergence reaches the set accuracy.

**Figure 4:** Variation of fitness curve when the genetic algorithm optimizes neural network.

**Figure 5:** Comparison between the output of different models and the expected output.

**Table 1:** Range of MASI reduction rate and treatment effect.

Treatment effect	MASI decline rate range
Basically healed	MASI decline rate ≥ 90%
Effective	MASI decline rate 50%~89%
Get better	MASI decline rate 10%~49%
Invalid	MASI decline rate < 10%

**Table 2:** Scoring criteria of each parameter of RCM.

Parameters	1	2	3	4
Epidermal pigmentation	<25.0%	26.0%-50.0%	51.0%-75.0%	76.0%-100%
Dendritic cells	None	≤5	≤15	>15
Melanophages	None	≤5	≤10	>10
Solar elastosis	Normal	Mild	Moderate	Serious
Vascularity	Normal	Mild	Moderate	Serious

**Table 3:** Validation results of the BP network model.

Sample	Expected output	BP model output	Error
1	0.151	0.125	0.024
2	0.243	0.273	0.033
3	0.060	0.092	0.032
4	0.192	0.214	0.024
5	0.533	0.483	0.046
6	0.582	0.561	0.018
7	0.422	0.442	0.022
8	0.3704	0.451	0.081
9	0.450	0.472	0.022
10	1.161	0.127	1.032

## Data Availability

The datasets used during the current study are available from the corresponding author on reasonable request.
